# Three Acupuncture Methods for Postoperative Pain in Mixed Hemorrhoids: A Systematic Review and Network Meta-Analysis

**DOI:** 10.1155/2022/5627550

**Published:** 2022-09-26

**Authors:** Sunsong Ye, Jianhua Zhou, Xiutian Guo, Xiaoxue Jiang

**Affiliations:** ^1^Department of Anorectology, Wenzhou Hospital of Traditional Chinese Medicine Affiliated to Zhejiang Chinese Medicine University, Wenzhou 325000, China; ^2^Department of Traditional Chinese Medicine, Shanghai Eighth People's Hospital, Shanghai 200235, China; ^3^Department of Anorectology, Shanghai Municipal Hospital of Traditional Chinese Medicine, Affiliated Shanghai University of Traditional Chinese Medicine, Shanghai 200071, China

## Abstract

**Background:**

Mixed hemorrhoids are a common anorectal disorder, surgery is the most effective means of eradicating hemorrhoids, and pain is the most common postoperative complication of mixed hemorrhoids.

**Objective:**

To compare the clinical efficacy of auricular plaster, acupoint application, and acupoint catgut embedding for treating postoperative pain in mixed hemorrhoids.

**Method:**

PubMed, Embase, The Cochrane Library, Web of Science, CNKI, Wanfang, VIP, and CBM databases were searched for randomized controlled trials (RCTs) of three acupuncture-related therapies for postoperative pain in mixed hemorrhoids from the time of database creation to October 2021. After screening the literature, extracting information, and evaluating the risk of bias of included studies, statistical analysis was performed using RevMan 5.3 and Stata 15.0.

**Result:**

Forty-seven RCTs with a total of 5121 patients were included. Network meta-analysis (NMA) showed that auricular plaster (OR = 5.90, 95% CI = (2.02, 17.21)) and acupoint catgut embedding therapy (OR = 5.55, 95% CI = (1.01, 30.40)) were more effective than analgesics in the treatment of postoperative pain in mixed hemorrhoids. The cumulative ranking probability (SUCRA) showed that acupoint application (73.6%) had the best overall efficacy and the rest were auricular plaster (68.7%), acupoint catgut embedding therapy (64.6%), auricular plaster combined with acupoint application (63.4%), and pain medication (8.9%) in that order. Secondly, auricular plaster (OR = −0.93, 95% CI = (−1.66, −0.20)), acupoint catgut embedding (OR = −0.8, 95% CI = (−1.50, −0.10)), and acupoint application (OR = −1.4, 95% CI = (−2.50, −0.31)) all led to a significant decrease in pain scores and were all more effective than analgesics. As ranked by SUCRA, the results showed that the efficacy of acupoint application (73.5%) was optimal and the rest were auricular plaster (56.1%), acupoint catgut embedding (50.2%), and pain medication (15.3%) in that order. In terms of pain degree, acupoint application (OR = 3.83, 95% CI = (1.25, 11.74)) was significantly better than pain medication.

**Conclusion:**

Acupoint application can improve the overall efficiency, reduce pain scores, and relieve the degree of postoperative pain in mixed hemorrhoids.

## 1. Introduction

Mixed hemorrhoids are a common anorectal disease [1], surgery is the most effective means of eradicating hemorrhoids [2], and pain is the most frequent postoperative complication of mixed hemorrhoids. Postoperative pain in hemorrhoids is a thorny problem that has troubled patients and physicians for a long time; it makes patients extremely nervous psychologically and fearful of defecation after surgery, which seriously affects the quality of surgery [3]. Pain arises for various reasons: (1) the innervation of the spinal nerve below the dentate line makes the pain response sensitive, (2) there is release of inflammatory mediators after surgery, and (3) there is postoperative stimulation of the wound surface by activities such as defecation and dressing changes, resulting in persistent spasm of the sphincter muscle [4].

In clinical practice, drug therapy is mostly used for postoperative pain in hemorrhoids but it requires multiple doses within a short period of time, which easily causes adverse reactions in the gastrointestinal tract and central nervous system, often resulting in dizziness, nausea, vomiting, dry mouth, and itchy skin [5–7], and the high cost of drugs increases the economic burden of patients. Therefore, the basic principle of pain management is to effectively relieve pain while minimizing the adverse effects of drugs and the cost of treatment. This has led to an urgent clinical need for nonpharmacological approaches to alleviate patients' pain and improve their quality of life.

Acupuncture is an important part of Traditional Chinese medicine, and acupuncture mainly includes auricular plaster, acupoint application, and acupoint catgut embedding, compared with conventional acupuncture, which is simple to operate, saves consumables and time cost, and can avoid the pain caused by applying regular acupuncture to patients. However, there is a lack of comparative studies on the efficacy of the three treatment methods and it is difficult to obtain a clear comparison by traditional meta-analysis. In this study, NMA was used to screen the best therapeutic measures based on ranking efficacy indexes for postoperative pain in hemorrhoid treatment in acupuncture to provide a reliable evidence-based reference for the clinic.

## 2. Methods and Analysis

### 2.1. Search Strategy

PubMed, Embase, The Cochrane Library, Web of Science, CNKI, Wanfang, VIP, and CBM databases were searched from the establishment to October 2021 to find clinical randomized controlled trials about 3 acupuncture therapies, auricular plaster, acupoint application, and acupoint catgut embedding, for the postoperation pain of mixed hemorrhoids. PubMed was used as an example, and a combination of subject terms and free words were used for the search. The search strategy is shown in Table 1.

#### 2.1.1. Inclusion Criteria

To be eligible for inclusion, the following criteria had to be fulfilled: (1) study design: RCTs; (2) study population: patients with postoperative pain in mixed hemorrhoids. Gender, age, and source of disease cases were not limited, and the mode of surgery and the degree of disease were not limited; (3) interventions: auricular plaster, acupoint application, and acupoint catgut embedding (can be one or more therapies combined) for the observation group and analgesic drugs or conventional treatment for the control group; (4) outcome indicators: the main indicators: (i) total effective rate, (ii) pain score, and (iii) pain degree; secondary indicators: (i) complications and (ii) adverse reactions; (5) efficacy evaluation criteria: (i) visual analog scoring VAS score, (ii) international standard pain assessment numerical grading method NRS, (iii) Changhai Pain Scale, (iv) WHO pain degree grading standard, divided into 0—III, and (v) numerical rating scale NRS score; and (6) Chinese Pain Society Han Jisheng recommended VAS.

#### 2.1.2. Exclusion Criteria

The following are the exclusion criteria: (1) study subjects: patients with combined postoperative pain from perianal diseases other than mixed hemorrhoids; (2) intervention: patients with combined herbal or proprietary Chinese medicine treatment; (3) experience, case reports, reviews, animal experiments, and case retrospective studies; (4) conference papers or dissertations, etc.; (5) repeatedly published literature; (6) outcome indicators: none or imperfect; and (7) the original text of the study not being obtained

### 2.2. Literature Screening

The retrieved literature records were managed using reference management software NoteExpress (version3.2). Based on the inclusion and exclusion criteria, two independent researchers conducted a detailed screening of titles and abstracts of reference records identified through database searching. All potential articles that meet the eligibility criteria and controversial literature were required for a full-text review. The third researcher will conduct the arbitration, who was responsible for resolving the conflict between the two researchers. A total of 924 relevant papers were obtained from the initial review, and 47 RCT studies were finally included after the stratified screening (Figure 1).

### 2.3. Quality Evaluation

Two investigators assessed the quality of the included studies according to the Cochrane Risk of Bias Assessment Tool recommended in the Cochrane Systematic Assessment Manual, version 5.1. The Cochrane Risk of Bias Assessment included seven aspects: randomization methods, blinding of participants and investigators, blinding of evaluators, allocation concealment, completeness of outcomes, selective reporting of outcomes, and other sources of bias. Bias was assessed for each of the included RCTs in terms of low risk, high risk, and unclear [8]. Any inconsistency was resolved through joint discussions with third-party investigators.

### 2.4. Data Information Collection

An Excel sheet database was set up to extract study information, including authors, year of publication, gender of study subjects, age, sample size, intervention measures, outcome indicators, complications, adverse events, surgical methods, and anesthesia methods.

### 2.5. Statistical Analysis

The risk bias was evaluated using RevMan 5.3 software. The included literature was compared directly using Stata 15.0 software, *I*^2^ ≤ 50%, *P* ≥ 0.05 was considered as no statistical heterogeneity in the included literature, and the meta-analysis was performed using the fixed-effect model; *I*^2^ > 50% or *P* < 0.05, the included literature was statistically heterogeneous, and a random-effects model was used for meta-analysis.

The ranking between interventions was obtained by direct and indirect comparisons using Stata 15.0 software, with odd ratios (OR) for dichotomous variables and standardized mean difference (SMD) and 95% credible intervals (CI) for continuous variables. The closed loop formed by studies with both direct and indirect evidence was performed to test inconsistency, the surface under the cumulative ranking curves (SUCRA) closer to 100%, the better the efficacy of the intervention, and the difference is considered statistically significant at *P* < 0.05.

## 3. Results

### 3.1. Results of Basic Characteristics of Included Studies and Risk of Bias Evaluation

A total of 5121 cases were included in 47 [7, 9–54] studies. A total of 47 RCTs were included in this study, of which 17 evaluated auricular plaster versus common treatment [10–14, 16, 18, 20, 21, 23, 24, 28, 29, 50–52, 54], 8 evaluated auricular plaster versus painkillers [15, 17, 22, 25–27, 30, 31], 5 evaluated acupoint catgut embedding versus common treatment [7, 34, 35, 37, 53], 7 evaluated acupoint catgut embedding versus painkillers [9, 36, 38, 39, 43–45], 6 evaluated acupoint application point versus common treatment [40–42, 47–49], 1 evaluated acupoint application point versus painkillers [33], 1 evaluated auricular plaster and acupoint application point versus painkillers [32], and 2 evaluated auricular plaster and acupoint application point versus common treatment [19, 46].

47 literature were all two-arm studies. 34 studies [7, 9–15, 17–19, 21–23, 28–31, 33–46, 48, 49] reported pain scores, 14 studies [9, 13, 16, 17, 19, 20, 22, 24–27, 39, 42, 47] reported the total efficiency, 9 studies [22, 26, 32, 42, 50–54] reported postoperative pain degree, and in terms of study design, 11 studies [11, 14, 17, 28, 29, 32, 33, 36, 43, 45, 46] reported adverse effects and detail management measures, 14 studies [11, 15, 17, 19, 34–36, 40, 42, 43, 46, 47, 52, 54] used random number tables, and 20 studies [9, 12, 18, 20–22, 26, 27, 29, 31–33, 37–39, 41, 45, 48, 50, 51] mentioned only the word random without details; 1 study [49] used randomization by lottery, 2 studies [23, 44] gave computerized random sequence, 2 studies [14, 30] used randomized block group design grouping, 3 studies [34, 36, 44] described case shedding, and 3 studies [7, 29, 48] used a blinded method. The basic characteristics of the included studies are shown in Table 2, and the results of the risk of bias evaluation are shown in Figures 2(a) and 2(b).

### 3.2. Direct Comparison Results of Meta-Analysis

#### 3.2.1. Total Effective Rate

A total of 14 studies reported the total effective rate, and the results of the meta-analysis showed that in terms of improving the total effective rate, auricular plaster combined with acupoint application (OR = 3.50, 95% CI (1.15, 10.63)), auricular plaster (OR = 8.06, 95% CI (4.80, 13.52)), and acupoint application (OR = 4.51, 95% CI (1.22, 16.61)) were superior to conventional treatment. Among the three, the efficacy of acupoint application was more significant (*P* < 0.05) (Figure 3). Acupoint catgut embedding (OR = 4.96, 95% CI (1.81, 13.54)) and auricular plaster (OR = 5.94, 95% CI (1.51, 23.46)) were superior to painkillers, and auricular plaster was more effective, with statistically significant differences (*P* < 0.05) (Figure 4).

#### 3.2.2. Pain Scoring

Auricular plaster (SMD = −1.92, 95%CI (−3.01, −0.83)), acupoint catgut embedding (SMD = −0.71, 95%CI (−0.95, −0.47)), and acupoint application (SMD = −1.35, 95%CI (−2.15, −0.55)) were better than conventional treatment, and auricular plaster was more effective (*P* < 0.05) (Figure 5). Acupoint catgut embedding (SMD = −1.06, 95%CI (−1.99, −0.13)), auricular plaster (SMD = −0.86, 95%CI (−1.38, −0.33)), and acupoint application (SMD = −6.39, 95%CI (−7.49, −5.30)) were all superior to pain medication, and the efficacy of acupoint application was statistically significant (*P* < 0.05) (Figure 6).

### 3.3. Results of Network Meta-Analysis (NMA)

#### 3.3.1. Network Evidence Diagram for Total Effective Rate, Pain Score, and Pain Degree

The total effective rate was included in 14 studies [9, 13, 16, 17, 19, 20, 22, 24–27, 39, 42, 47] and pain degree in 9 studies [22, 26, 32, 42, 50–54], both without closed loop formation (Figures 7(a) and 7(b)).

A total of 34 papers [7, 9–15, 17–19, 21–23, 28–31, 33–46, 48, 49] were included in the pain score, involving 6 treatment measures (auricular plaster, acupoint catgut embedding, acupoint application, conventional treatment, and pain medication), forming a total of 3 closed loops, namely, conventional treatment-acupoint application-painkiller-acupoint catgut embedding, conventional treatment-acupoint application-painkiller-auricular plaster, and conventional treatment-acupoint catgut embedding-painkiller-auricular plaster (Figure 7(c)).

#### 3.3.2. Total Efficiency

In terms of improving the total effective rate, auricular plaster (OR = 5.90, 95%CI = (2.02, 17.21)) and acupoint catgut embedding (OR = 5.55, 95%CI = (1.01, 30.40)) had higher total efficiency than painkillers. Auricular plaster (OR = 3.66, 95%CI = (1.33, 10.13)) was superior than conventional treatment, and the differences were all statistically significant, *P* < 0.05 (Table 3 and Figure 8(a)).

The efficacy ranking was based on cumulative SUCRA, and the larger the area, the better the efficacy. The results of SUCRA ranking showed that acupoint application (73.6%) > auricular plaster (68.7%) > acupoint catgut embedding (64.6%) > auricular plaster combined with acupoint application (63.4%) > conventional treatment (20.9%) > painkillers (8.9%) (Table 4 and Figure 8(b)).

#### 3.3.3. Pain Scoring

In terms of pain score reduction, auricular plaster (OR = −0.93, 95%CI = (−1.66, −0.20)), acupoint catgut embedding (OR = −0.8, 95%CI = (−1.50, −0.10)), and acupoint application (OR = −1.4, 95%CI = (−2.50, −0.31)) were superior to painkillers. Auricular plaster (OR = −1.20, 95%CI = (−1.86, −0.55)), acupoint catgut embedding (OR = −1.07, 95%CI = (−1.85, −0.29)), and acupoint application (OR = −1.68, 95%CI = (−2.56, −0.79)) were superior to conventional treatment.

Auricular plaster combined with acupoint application was superior to auricular plaster (OR = −3.27, 95%CI = (−5.70, −0.84)), acupoint catgut embedding (OR = −3.41, 95%CI = (−5.86, −0.95)), acupoint application (OR = −2.80, 95%CI = (−5.28, −0.33)), conventional treatment (OR = −4.48, 95%CI = (−6.81, −2.15)), and painkillers (OR = −4.20, 95%CI = (−6.67, −1.74)); all differences were statistically significant, *P* < 0.05 (Table 5 and Figure 9(a)).

The results of the area under the curve (SUCRA) ranking showed that auricular plaster combined with acupoint application (99.5%) > acupoint application (73.5%) > auricular plaster (56.1%) > acupoint catgut embedding therapy (50.2%) > pain medication (15.3%) > conventional treatment (5.3%) (Table 6 and Figure 9(b)).

#### 3.3.4. Pain Degree

After treatment, patients with no pain and mild pain were significantly relieved but there was no significant effect on the symptoms of patients with moderate and severe pain. The results showed that auricular plaster (OR = 3.13, 95%CI = (2.00, 4.89)) and acupoint application (OR = 6.18, 95%CI = (3.11, 12.28)) were better than conventional treatment and acupoint application (OR = 3.83, 95%CI = (1.25, 11.74)) was better than painkillers; all differences were statistically significant, *P* < 0.05 (Table 7 and Figure 10(a)).

The results of the area under the curve (SUCRA) ranking showed that acupoint application (91.2%) > auricular plaster (66.1%) > auricular plaster combined with acupoint application (54.6%) > painkillers(36.6%) > acupoint catgut embedding (34.8%) > conventional treatment (16.8%); all differences were statistically significant, *P* < 0.05 (Table 8 and Figure 10(b)).

#### 3.3.5. Complications and Adverse Reactions

Six publications reported complications [31, 33, 36, 37, 44, 53] in a total of 490 patients, of which 133 patients developed complications. In terms of reducing postoperative complications, auricular plaster (RR = 0.24, 95%CI = (0.06, 0.96)) and acupoint catgut embedding (RR = 0.28, 95% = CI (0.12, 0.69)) were superior to painkillers and auricular plaster (RR = 0.15, 95%CI = (0.03, 0.89)) and acupoint catgut embedding (RR = 0.18, 95% = CI (0.10,0.33)) were superior to conventional treatment and the differences were statistically significant, *P* < 0.05 (Table 9 and Figure 11(a)).

The results of SUCRA ranking showed that acupoint application (86.5%) > auricular plaster (69.6%) > acupoint catgut embedding (65.8%) > painkillers(21.5%) > conventional treatment (6.6%) (Figure 11(b)). Regarding adverse reactions, a total of 10 publications reported [11, 14, 17, 28, 29, 32, 33, 36, 43, 45, 46] a total of 844 patients, of which 100 patients experienced adverse reactions. In terms of reducing patients' adverse reactions, auricular plaster (RR = 0.2, 95%CI = (0.04, 0.97)), acupoint catgut embedding (RR = 0.04, 95%CI = (0.01, 0.21)), and auricular plaster combined with acupoint application (RR = 0.19, 95%CI = (0.05, 0.69)) were superior to conventional treatment and auricular plaster (RR = 0.15, 95%CI = (0.05, 0.48)), acupoint catgut embedding (RR = 0.03, 95%CI = (0.01, 0.11)), and auricular plaster combined with acupoint application (RR = 0.14, 95%CI = (0.02, 0.83)) were superior to painkillers and the differences were statistically significant, *P* < 0.05 (Table 10 and Figure 12(a)). The results of SUCRA ranking showed that acupoint catgut embedding (96.2%) > auricular plaster combined with acupoint application (64.9%) > auricular plaster (63%) > acupoint application (43.5%) > conventional treatment (20.3%) > painkillers (12.2%) (Figure 12(b)).

#### 3.3.6. Duration of Onset of Acupuncture Intervention

Meta-analysis results showed that the control group was conventional treatment; 24 h after intervention treatment, SMD = −1.40, 95%CI = (−2.05, −0.74), 48 h, SMD = −1.14, 95%CI = (−1.55, −0.74), and 72 h, SMD = −1.80, 95%CI = (−2.48, −1.11) all played a pain relief effect, with the 72 h efficacy being more effective. In the control group with analgesics, 24 h, SMD = −1.33, 95%CI = (−2.07, −0.60), 48 h, SMD = −1.33, 95%CI = (−2.27, −0.40), and 72 h, SMD = −2.12, 95%CI = (−3.21, −1.03) after the intervention had an analgesic effect, the efficacy of 72 h was more visible, and all differences were statistically significant, *P* < 0.05 (Figures 13(a) and 13(b)).

## 4. Publication Bias Analysis and Small Sample Effect Assessment

Because 34 of the 47 publications reported pain scores, this study used pain scores as an outcome indicator to test for small sample effects or publication bias and the funnel plot showed that most of the study scatters were located between the funnel plot and were more symmetrical, suggesting that there may be a small publication bias (Figure 14).

## 5. Discussion

This study is aimed at discussing the efficacy of three different acupuncture therapies (auricular plaster, acupoint application, and acupoint catgut embedding) for postoperative pain in mixed hemorrhoids. 47 RCTs involving 5121 patients were included in this study. The results of the NMA showed that auricular plaster, acupoint application, and acupoint catgut embedding were superior to pain medication and conventional treatment in improving the overall efficiency and the ranking results showed that acupoint application was the most effective. Reducing postoperative pain scores, auricular plaster, acupoint application, and acupoint catgut embedding were superior to pain medication and conventional treatment. Auricular plaster combined with acupoint application was probably the most effective, followed by acupoint application.

However, of the 47 studies included in this study, only 3 [19, 32, 46] had auricular plaster combined with acupoint application, which is a small sample size, and more studies need to be included to confirm the efficacy of the combined therapy. In terms of reducing postoperative complications, auricular plaster, acupoint application, and acupoint catgut embedding were superior to pain medication and conventional treatment and acupoint application was the most effective, significantly reducing postoperative edema, urinary retention, and other complications; in terms of safety, auricular plaster, acupoint application, and acupoint catgut embedding were superior to pain medication. Acupoint catgut embedding was the most effective for the onset of effect of the three acupuncture interventions; it was found that the analgesic effect was superior to that of analgesics at different time periods of 24 h, 48 h, and 72 h postoperatively. The perianal area is a concentrated area of nerve endings and is more sensitive to nociception. As the effects of anesthesia wear off, patients have a painful process that lasts 24 h to 48 h [55]. This study found that it still has a better analgesic effect at 72 h postoperatively, indicating that the effect of acupuncture for postoperative pain on mixed hemorrhoids is long lasting and stable, guiding that the treatment course of the three acupuncture therapies for postoperative pain in mixed hemorrhoids should last at least until 72 h for better therapeutic effect.

Nowadays, medical treatment of postoperative pain in mixed hemorrhoids mostly uses opioid analgesics, nonsteroidal anti-inflammatory drugs, central analgesics, etc. Although the pain relief effect is good, drug side effects such as nausea, dizziness, vomiting, and sweating can easily occur [56, 57], with adverse reactions as high as 37% [58]. Acupuncture therapy, as a green complementary alternative therapy, has better clinical efficacy for postoperative pain in mixed hemorrhoids.

This study showed that the efficacy of acupoint application for postoperative pain in mixed hemorrhoids was more advantageous compared with other therapies. In fact, the mechanism of acupoint application for postoperative pain in mixed hemorrhoids is more widely studied, which may be related to its good efficacy. Acupoint application is based on the guidance of Chinese medicine meridian science, and the drug is applied to specific points on the body surface, both for acupuncture point stimulation and for absorbing the active ingredients of the drug through the skin tissue, producing a local concentration of the drug and playing the dual role of Chinese medicine and meridian regulation at the same time. Medical research has shown that trans-acupoint application drugs have permeability, exosensitivity, and amplification effects [59].

This study showed that the efficacy of acupoint application for postoperative pain in mixed hemorrhoids was more advantageous compared with other therapies. In fact, the mechanism of acupoint application for postoperative pain in mixed hemorrhoids is more widely studied, which may be related to its good efficacy. Acupoint application is based on the guidance of Chinese medicine meridian science. The drug is applied to specific points on the body surface, both for acupuncture point stimulation and for absorbing the active ingredients of the drug through the skin tissue, producing a local concentration of the drug and playing the dual role of Chinese medicine and meridian regulation at the same time. Medical research has shown that trans-acupoint-applied drugs have permeability, exosensitivity, and amplification effects [47]. Another study showed that acupoint application could produce the effect of biological function through biological wave meridian points, through the process of absorption, transmission, and reflection, to activate blood and remove blood stasis, unblock meridians, and achieve pain relief [59]. The local absorption of drugs in the skin reduces the adverse reactions in the gastrointestinal tract [60]. In modern medicine, acupoint application therapy is classified as TDS, the transdermal drug delivery system of Chinese medicine [61]. 90% of the human dermis is a vascular-rich connective tissue, and the drug is absorbed into the blood through keratin transit, and the keratin layer is the main barrier for transdermal absorption, which forms a dense state locally after acupoint application, causing the cells of the keratin layer to swell into a porous state and make its tight structure lose, letting it easy for the drug to penetrate [62].

As a part of Chinese traditional medicine, acupuncture therapy has the advantages of precise efficacy, low toxic side effects, and easy acceptance by patients. In recent years, acupuncture therapy has gradually become the mainstream of global medicine as a green alternative or complementary treatment [63, 64]. Compared with conventional drug therapy, it can effectively reduce drug side effects and postoperative complications such as urinary retention and traumatic edema, as well as reduce the economic burden of patients [65, 66], and even if it cannot completely replace analgesics, it can participate in the synergistic use of drugs and reduce the number and dose of analgesic drugs taken by patients, thus reducing the occurrence of adverse reactions in patients. Compared to ordinary acupuncture, the three acupuncture treatments avoid the pain caused to patients by multiple needle sticks, reduce the workload of medical personnel, and make up for the short duration of the curative effect of ordinary acupuncture and the large arbitrariness of the operation. More importantly, there is no need to change the needles daily, which helps improve patient compliance and promote the clinical grassroot application.

This study still has shortcomings, such as the lack of systematic and standardized methods for making homemade acupoint-applied plasters and the need to further standardize the methods for making acupoint-applied plasters. The methodological quality of the included studies was low, most of the studies did not mention the distribution concealment method, and due to the specificity of acupuncture therapy, most of the studies were not implemented blinded, which may produce implementation bias; in order to reduce bias and make the results more reliable, in the future, researchers should follow the CONSORT reporting standards [67]. The control group has drug interventions which did not consider the drug dose and duration and frequency, and the specific content of the acupuncture protocol was not explored, such as TCM identification, treatment frequency, and duration; the details of acupuncture therapy were reported unclear, which to some extent caused the bias of the study results and decreased the guiding effect on TCM clinical practice, and in future studies, clinical trials of acupuncture therapy should follow STRICTA standards [68]. For combination therapy, there are fewer clinical research trials, which can be a focus of future research to provide more possibilities for the selection of analgesic methods and provide evidence-based medical evidence reference for the use of this method in clinical practice. In a word, given the very low methodological quality of the included systematic evaluations and the risk bias of poor reporting of randomized controlled trials, a more rigorous design and standardized reporting are needed in the future to demonstrate the reliability of this study further.

## 6. Conclusion

Current evidence suggests that acupoint application therapy for the treatment of postoperative pain in mixed hemorrhoids has better efficacy in improving overall effectiveness and reducing pain scores as well as relieving pain levels.

## Figures and Tables

**Figure 1:** Flow chart literature screening.

**Figure 2:** Results of basic characteristics of included studies and risk of bias evaluation. (a) Risk of bias graph. (b) Risk of bias summary.

**Figure 3:** Forest plot of meta-analysis of the overall efficacy of three different acupuncture methods for postoperative pain relief of mixed hemorrhoids (compared with conventional treatment).

**Figure 4:** Forest plot of meta-analysis of the overall efficacy of three different acupuncture methods for postoperative pain relief of mixed hemorrhoids (compared with analgesics).

**Figure 5:** Forest map of meta-analysis of three acupuncture methods for postoperative pain scores of mixed hemorrhoids (compared with conventional treatment).

**Figure 6:** Forest map of meta-analysis of three acupuncture methods for postoperative pain scores of mixed hemorrhoids (compared with analgesics).

**Figure 7:** Network evidence diagram for the total effective rate, pain score, and pain degree. (a) Total effective rate evidence network diagram. (b) Network diagram of evidence of the pain degree. (c) Pain score evidence network diagram.

**Figure 8:** Total efficiency. (a) Forest map of different treatment methods of the total effective rate for mixed hemorrhoids. (b) Sucra diagram of the total effective rate of different methods for postoperative pain.

**Figure 9:** Pain scoring. (a) Forest map of the pain score after different treatment methods. (b) Sucra plot of the pain score after different treatment methods.

**Figure 10:** Pain degree. (a) Forest map of the pain degree after different treatment methods. (b) Sucra diagram of the pain degree after different methods for postoperative pain.

**Figure 11:** Complications. (a) Forest map of complications after the treatment of postoperative pain by different methods. (b) Sucra diagram of complication after the treatment of postoperative pain by different methods.

**Figure 12:** Adverse reactions. (a) Forest map of adverse reactions after the treatment of postoperative pain by different methods. (b) Sucra diagram of adverse reactions after the treatment of postoperative pain by different methods.

**Figure 13:** Duration of onset of acupuncture intervention. (a, b) Meta-analysis of postoperative pain scores of mixed hemorrhoids treated with acupuncture at different times.

**Figure 14:** Comparison of different acupuncture in treating postoperative pain of mixed hemorrhoids by adjusting the funnel plot.

**Table 1:** Search strategy in PubMed.

Search	Query
#1 Search: (“Acupuncture”[Mesh]) OR (Auricular point[Title/Abstract]) OR (Auricular plaster therapy[Title/Abstract]) OR (acupoint catgut embedding[Title/Abstract]) OR (acupoint application therapy[Title/Abstract]) #2 Search: (“hemorrhoidectomy” [Mesh]) OR ((postoperative pain of mixed hemorrhoids [Title/Abstract]) OR (hemorrhoid excision[Title/Abstract]) OR (hemorrhoid surgery acupuncture [Title/Abstract]) #3 Search: randomized controlled trial[Publication Type] OR randomized[Title/Abstract] OR placebo[Title/Abstract] #4 Search: #1 and #2 and #3	

**Table 2:** The basic characteristics of the included studies.

Author year	Sample size	Treatment group 1	Treatment group 2	Anesthetic mode	Operation method	Outcome	Adverse reactions and complications
		Intervention age (year)/course (year)	Intervention age (year)/course (year)				
Xiong and Xie [9]	63	Acupoint catgut embedding therapy 41.1 ± 13.5/9.7 ± 4.1	Analgesic 43.1 ± 13.7/10.3 ± 4.6	NA	NA	1, 2	NA
Chen and Deng [10]	40	Auricular plaster 45.5 ± 23.5/NA	Regular treatment 45.0 ± 22.0/NA	NA	NA	2	NA
Fang et al. [11]	66	Auricular plaster 38.7 ± 10.5/NA	Regular treatment 40.8 ± 11.8/NA	NA	NA	3	Treatment group 1: none; treatment group 2: 1 case of perianal skin pruritus and wound bleeding, 1 case of asthma, and 1 case of abnormal liver function and urinary tract infection
Zhu et al. [12]	120	Auricular plaster 37.4/NA	Regular treatment 37.8/NA	Lumbar anesthesia	MM	1	NA
Huang et al. [13]	120	Auricular plaster 38/NA	Regular treatment 38/NA	Lumbar anesthesia	MM	1, 2	NA
Di et al. [14]	60	Auricular plaster 42.93 ± 10.94/NA	Regular treatment 45.69 ± 9.07/NA	Lumbar anesthesia	PPH	2	Treatment group 1: 1 case of dizziness and 2 cases of dry mouth, 3 cases of dizziness; treatment group 2: 2 cases of nausea, 1 case of vomiting, and 3 cases of dry mouth
Gao and Liu [15]	90	Auricular plaster 44.58 ± 10.98/NA	Analgesic 42.17 ± 11.5/NA	NA	MM	3	NA
Liu and Zheng [16]	601	Auricular plaster NA/NA	Regular treatment NA/NA	Local anesthesia	MM	1	NA
Di et al. [17]	120	Auricular plaster 45.15 ± 2.53/NA	Analgesic 47.08 ± 3.09/NA	Lumbar anesthesia	PPH	1	Treatment group 1: none; treatment group 2: 2 cases of dizziness, 3 cases of nausea, 1 case of vomiting, 1 case of drowsiness, and 1 case of dry mouth
Yan [18]	120	Auricular plaster NA/NA	Regular treatment NA/NA	Local anesthesia	MM	2	NA
Yang et al. [19]	100	Auricular plaster combined with acupoint application 41.5 ± 3.5/15.1 ± 5.6	Regular treatment 40.2 ± 2.6/14.9 ± 6.8	NA	NA	1, 2	NA
Hu [20]	120	Auricular plaster 34/NA	Regular treatment 33/NA	NA	NA	1	NA
Liu et al. [21]	140	Auricular plaster 47.5 ± 5.6/NA	Regular treatment 48.8 ± 6.4/NA	NA	NA	2	NA
Beilei et al. [22]	66	Auricular plaster 46.52 ± 3.71/4.03 ± 2.87	Analgesic 45.92 ± 3.63/4.06 ± 2.91	NA	NA	1, 2, 3	NA
Chen et al. [23]	224	Auricular plaster 50.1 ± 8.2/NA	Regular treatment 51.6 ± 9.0/NA	NA	MM	3	NA
Gan [24]	271	Auricular plaster NA/NA	Regular treatment NA/NA	Lumbar anesthesia	MM	1	NA
Tang and Hu [25]	40	Auricular plaster 31/NA	Analgesic 31/NA	Lumbar anesthesia	MM	1	NA
Hong et al. [26]	100	Auricular plaster 60/NA	Analgesic 58/NA	Local anesthesia	MM	1, 3	NA
Chai and Feng [27]	140	Auricular plaster 41.87/NA	Analgesic 42.13/NA	NA	NA	1	NA
Yang [28]	60	Auricular plaster 38.06 ± 3.52/NA	Regular treatment 37.52 ± 3.64/NA	NA	NA	2	Treatment group 1: none; treatment group 2: 2 cases of dizziness, 1 case of chest tightness, and 1 case of urticaria
Zhang [29]	60	Auricular plaster 34.55 ± 3.63/10.48 ± 1.35	Regular treatment 39.22 ± 1.56/11.12 ± 1.82	NA	NA	3	None
Li [30]	106	Auricular plaster 42.9 ± 7.0/NA	Analgesic 42.7 ± 7.1/NA	NA	NA	1	NA
Pan [31]	80	Auricular plaster 48.50 ± 5.75/3.68 ± 0.55	Analgesic 47.50 ± 5.63/3.50 ± 0.68	NA	NA	2	Treatment group 1: 2 cases with irregular defecation and 1 case with edema; treatment group 2: 4 cases of urinary retention, 1 case of bleeding, 2 cases of irregular defecation, and 3 cases of edema
Zheng and Yv [32]	120	Auricular plaster combined with acupoint application 37.2 ± 7.2/NA	Analgesic 35.3 ± 8.5/NA	NA	NA	3	Treatment group 1: none; treatment group 2: 7 cases with mild stomach pain and other stomach upset symptoms
Wang and Chen [33]	80	Acupoint application 32.15 ± 10.12/NA	Analgesic 33.85 ± 9.96/NA	NA	MM	2	Treatment group 1: none; treatment group 2: postoperative urinary retention in 3 cases, local trauma tissue edema in 2 cases; postoperative stomachache was relieved spontaneously in 1 case
Huang et al. [34]	60	Acupoint catgut embedding therapy 41.2 ± 10.05/NA	Regular treatment 42.3 ± 11.7/NA	Local anesthesia	MM	2	NA
Li et al. [35]	120	Acupoint catgut embedding therapy 41.2 ± 10.5/10.1 ± 0.5	Regular treatment 42.3 ± 11.7/9.2 ± 0.4	Caudal anesthesia	MM	3	NA
Yang et al. [36]	120	Acupoint catgut embedding therapy 42.1 ± 11.5/NA	Analgesic 43.6 ± 12.1/NA	Local anesthesia	MM	2	Treatment group 1: 2 cases of urinary retention, 7 cases of edema, and 1 case of nausea; treatment group 2: 8 cases of urinary retention, 17 cases of edema, 6 cases of nausea, 4 cases of vomiting, and 5 cases of vertigo
Sheng et al. [37]	60	Acupoint catgut embedding therapy 43 ± 16/NA	Regular treatment 44 ± 15/NA	Lumbar anesthesia	MM	2	Treatment group 1: 3 cases of irregular defecation and 2 cases of anal edema; treatment group 2: 10 cases of irregular defecation and 8 cases of anal edema
Yue and Li [38]	200	Acupoint catgut embedding therapy 46.5/NA	Analgesic 47.3/NA	NA	MM	1	NA
Zhang [39]	70	Acupoint catgut embedding therapy 35 ± 10/2.9 ± 1.4	Analgesic 34 ± 12/13.1 ± 1.2	NA	NA	2	NA
Liang et al. [40]	60	Acupoint application	Regular treatment	NA	MM	2	NA
Li [41]	30	Acupoint application	Regular treatment	NA	NA	3	NA
Meng et al. [42]	160	Acupoint application	Regular treatment	NA	NA	1, 2, 3	NA
Zhou et al. [43]	90	Acupoint catgut embedding therapy 36 ± 4/7.8 ± 2.1	Analgesic 35 ± 7/7.3 ± 2.00	CSEA	MM	2	Treatment group 1: 1 case of nausea and vomiting, 1 case of localized skin discomfort; treatment group 2: 8 cases of dizziness and headache, 13 cases of nausea and vomiting, 6 cases of being flustered, and 4 cases of local skin discomfort
Li et al. [44]	90	Acupoint catgut embedding therapy 44.9 ± 5.7/9.3 ± 0.2	Analgesic 46.4 ± 4.9/10.5 ± 0.4	Local anesthesia	MM	3	Treatment group 1: 7 cases had difficulty urinating and 4 cases had edema; treatment group 2: 15 cases had difficulty urinating and 9 cases had edema
Du [45]	60	Acupoint catgut embedding therapy 41.3 ± 12.08/4.88 ± 3.12	Analgesic 42.88 ± 11.93/5.79 ± 2.64	Local anesthesia	MM	2	Treatment group 1: none; treatment group 2: 3 cases of nausea and vomiting
Wang [46]	68	Auricular plaster combined with acupoint application 45.58 ± 11.98/NA	Regular treatment 43.17 ± 12.5/NA	Lumbar anesthesia	MM	2	Treatment group 1: 2 cases of nausea, 1 case of vomiting; treatment group 2: 5 cases of nausea, 3 cases of vomiting, 1 case of stomatitis, 1 case of allergic dermatitis
Liang and Wen [47]	96	Acupoint application 60.10 ± 8.23/NA	Regular treatment 58.23 ± 8.97/NA	Intravertebral canal anesthesia	MM	1	NA
Wang et al. [48]	90	Acupoint application 48.8 ± 12.6/NA	Regular treatment 43.2 ± 14.0/NA	NA	NA	1	NA
Xie and Huang [49]	60	Acupoint application 47.1 ± 4.6/NA	Regular treatment 46.2 ± 4.3/NA	Local anesthesia	MM	2	NA
Huang et al. [50]	60	Auricular plaster 42.1 ± 8.52/NA	Regular treatment 41.3 ± 10.37/NA	Local anesthesia	MM	2	None
Ma [51]	150	Auricular plaster 41.7 ± 0.7/3.2 ± 0.3	Regular treatment 42.6 ± 0.5/3.1 ± 0.5	NA	NA	1	NA
Sun and Chen [52]	100	Auricular plaster	Regular treatment	NA	MM	2	NA
Wang et al. [53]	60	Acupoint catgut embedding therapy 40 ± 6.64/NA	Regular treatment 38 ± 7.02/NA	Intravertebral canal anesthesia	NA	3	Treatment group 1: 3 cases of voiding difficulties and 2 cases of edema; treatment group 2: 10 cases of voiding difficulties, 8 cases of edema
Yan et al. [54]	80	Auricular plaster 41.39 ± 9.4/NA	Regular treatment 46.18 ± 13.18/NA	NA	NA	3	NA
Pei et al. [7]	130	Acupoint catgut embedding therapy	Regular treatment	NA	MM	2	NA

Outcome indicators: 1: total effective rate; 2: pain score; 3: pain degree; NA: not available; MM: Milligan-Morgan; PPH: procedure for prolapse and hemorrhoids; CSEA: combined spinal-epidural anesthesia.

**Table 3:** Network meta-analysis of the overall efficacy of different treatment therapies (OR (95% CI)].

Acupoint application	0.77 (0.09, 6.33)	0.73 (0.04, 13.34)	0.74 (0.04, 12.22)	0.21 (0.03, 1.33)	0.13 (0.01, 1.39)
1.29 (0.16, 10.54)	Auricular	Point 0.94 (0.13, 7.02)	0.96 (0.09, 10.01)	0.27 (0.10, 0.75)	0.17 (0.06, 0.49)
1.37 (0.07, 25.04)	1.06 (0.14, 7.91)	Acupoint catgut embedding	1.01 (0.05, 22.31)	0.29 (0.03, 2.75)	0.18 (0.03, 0.99)
1.35 (0.08, 22.31)	1.05 (0.10, 10.97)	0.99 (0.04, 21.69)	Auricular point and acupoint application	0.29 (0.03, 2.38)	0.18 (0.01, 2.35)
4.73 (0.75, 29.71)	3.66 (1.33, 10.13)	3.45 (0.36, 32.79)	3.50 (0.42, 29.10)	Regular treatment	0.62 (0.14, 2.72)
7.61 (0.72, 80.39)	5.90 (2.02, 17.21)	5.55 (1.01, 30.40)	5.63 (0.43, 74.46)	1.61 (0.37, 7.04)	Analgesic drugs

**Table 4:** Sucra ratio of total effective rate of different treatment methods.

Treatment	SUCRA	PrBest	MeanRank
Auricular point	68.7	12.5	2.6
Acupoint catgut embedding	64.6	25.6	2.8
Acupoint application	73.6	36.1	2.3
Regular treatment	20.9	0.0	5.0
Analgesic drugs	8.9	0.0	5.6
Auricular point and acupoint application	63.4	25.9	2.8

**Table 5:** Network meta-analysis of the pain score of different treatment therapies (SMD (95% CI)).

Auricular point and acupoint application	2.80 (0.33, 5.28)	3.27 (0.84, 5.70)	3.41 (0.95, 5.86)	4.20 (1.74, 6.67)	4.48 (2.15, 6.81)
−2.80 (−5.28, −0.33)	Acupoint application	0.47 (−0.59, 1.53)	0.60 (−0.52, 1.73)	1.40 (0.31, 2.50)	1.68 (0.79, 2.56)
−3.27 (−5.70, −0.84)	−0.47 (−1.53, 0.59)	Auricular point	0.13 (−0.72, 0.98)	0.93 (0.20, 1.66)	1.20 (0.55, 1.86)
−3.41 (−5.86, −0.95)	−0.60 (−1.73, 0.52)	−0.13 (−0.98, 0.72)	Acupoint catgut embedding	0.80 (0.10, 1.50)	1.07 (0.29, 1.85)
−4.20 (−6.67, −1.74)	−1.40 (−2.50, −0.31)	−0.93 (−1.66, −0.20)	−0.80 (−1.50, −0.10)	Analgesic drugs	0.27 (−0.52, 1.07)
−4.48 (−6.81, −2.15)	−1.68 (−2.56, −0.79)	−1.20 (−1.86, −0.55)	−1.07 (−1.85, −0.29)	−0.27 (−1.07, 0.52)	Regular treatment

**Table 6:** Sucra proportion table of the pain score of different treatment methods.

Treatment	SUCRA	PrBest	MeanRank
Auricular point	56.1	0.1	3.2
Acupoint catgut embedding	50.2	0.1	3.5
Acupoint application	73.5	1.3	2.3
Regular treatment	5.3	0.0	5.7
Analgesic drugs	15.3	0.0	5.2
Auricular point and acupoint application	99.5	98.5	1.0

**Table 7:** Network meta-analysis of the pain degree of patients with mixed hemorrhoids treated by different methods (OR (95% CI)).

Acupoint application	0.51 (0.22, 1.15)	0.40 (0.05, 3.40)	0.26 (0.09, 0.80)	0.16 (0.00, 8.93)	0.16 (0.08, 0.32)
1.98 (0.87, 4.48)	Auricular point	0.79 (0.11, 5.71)	0.52 (0.24, 1.11)	0.32 (0.01, 17.06)	0.32 (0.20, 0.50)
2.51 (0.29, 21.36)	1.27 (0.18, 9.18)	Auricular point and acupoint application	0.66 (0.11, 4.07)	0.41 (0.00, 34.47)	0.41 (0.05, 3.09)
3.83 (1.25, 11.74)	1.94 (0.90, 4.16)	1.53 (0.25, 9.48)	Analgesic drugs	0.62 (0.01, 35.52)	0.62 (0.26, 1.50)
6.18 (0.11, 340.82)	3.13 (0.06, 166.63)	2.46 (0.03, 209.31)	1.61 (0.03, 92.59)	Acupoint catgut embedding	1.00 (0.02, 51.97)
6.18 (3.11, 12.28)	3.13 (2.00, 4.89)	2.47 (0.32, 18.76)	1.62 (0.67, 3.92)	1.00 (0.02, 52.02)	Regular treatment

**Table 8:** Sucra proportion table of the pain degree in patients with mixed hemorrhoids treated by different methods.

Treatment	SUCRA	PrBest	MeanRank
Auricular point	66.1	1.9	2.7
Acupoint catgut embedding	34.8	17.3	4.3
Acupoint catgut embedding	91.2	63.8	1.4
Regular treatment	16.8	0	5.2
Analgesic drugs	36.6	0.2	4.2
Auricular point and acupoint application	54.6	16.7	3.3

**Table 9:** Network meta-analysis of complications that occurred in patients with mixed hemorrhoids treated by different methods (RR (95% CI)).

Acupoint application	3.05 (0.12, 77.68)	3.55 (0.17, 76.05)	12.55 (0.67, 234.86)	19.72 (0.87, 448.52)
0.33 (0.01, 8.34)	Auricular point	1.16 (0.22, 6.02)	4.11 (1.04, 16.29)	6.46 (1.12, 37.31)
0.28 (0.01, 6.03)	0.86 (0.17, 4.44)	Acupoint catgut embedding	3.53 (1.44, 8.67)	5.55 (3.01, 10.23)
0.08 (0.00, 1.49)	0.24 (0.06, 0.96)	0.28 (0.12, 0.69)	Analgesic drugs	1.57 (0.53, 4.65)
0.05 (0.00, 1.15)	0.15 (0.03, 0.89)	0.18 (0.10, 0.33)	0.64 (0.21, 1.88)	Regular treatment

**Table 10:** Network meta-analysis of adverse reaction that occurred in patients with mixed hemorrhoids treated by different methods (RR (95% CI)).

Acupoint catgut embedding	4.30 (0.67, 27.82)	4.57 (0.94, 22.30)	9.91 (0.31, 315.19)	22.72 (4.77, 108.27)	30.48 (8.81, 105.38)
0.23 (0.04, 1.50)	Auricular point and acupoint application	1.06 (0.17, 6.84)	2.30 (0.06, 91.53)	5.28 (1.45, 19.18)	7.08 (1.21, 41.53)
0.22 (0.04, 1.07)	0.94 (0.15, 6.06)	Auricular point	2.17 (0.07, 67.20)	4.97 (1.04, 23.82)	6.67 (2.07, 21.43)
0.10 (0.00, 3.21)	0.43 (0.01, 17.26)	0.46 (0.01, 14.32)	Acupoint application	2.29 (0.06, 81.97)	3.08 (0.12, 77.78)
0.04 (0.01, 0.21)	0.19 (0.05, 0.69)	0.20 (0.04, 0.97)	0.44 (0.01, 15.59)	Regular treatment	1.34 (0.29, 6.23)
0.03 (0.01, 0.11)	0.14 (0.02, 0.83)	0.15 (0.05, 0.48)	0.33 (0.01, 8.22)	0.75 (0.16, 3.46)	Analgesic drugs

## Data Availability

The datasets used and/or analyzed during the current study are available from the corresponding author upon reasonable request.
